# Aconitine Induces TRPV2-Mediated Ca^2+^ Influx through the p38 MAPK Signal and Promotes Cardiomyocyte Apoptosis

**DOI:** 10.1155/2021/9567056

**Published:** 2021-09-01

**Authors:** Chunai Yang, Xiaoyan Zeng, Zhongfeng Cheng, Junbo Zhu, Yangshan Fu

**Affiliations:** ^1^Department of Emergency, The Affiliated Hospital of Yunnan University, Kunming 650021, China; ^2^Department of the Teaching Office, School of Continuing Education, Kunming Medical University, Kunming 650500, China

## Abstract

Aconitine is the main effective component of traditional Chinese medicine *Aconitum*, which has been proved to have severe cardiovascular toxicity. The toxic effect of aconitine on cardiomyocytes is related to intracellular calcium overload, but the mechanism remains unclear. The aim of this study was to explore the mechanism of aconitine inducing intracellular Ca^2+^ overload and promoting H9c2 cardiomyocyte apoptosis through transient receptor potential cation channel subfamily V member 2 (TRPV2). After treated with different concentrations of aconitine, the level of cell apoptosis, intracellular Ca^2+^, and expression of p-p38 MAPK and TRPV2 of H9c2 cardiomyocytes were detected. The results showed that aconitine induced Ca^2+^ influx and H9c2 cardiomyocyte apoptosis in a dose-dependent manner and promoted p38 MAPK activation as well as TRPV2 expression and plasma membrane (PM) metastasis. siTRPV2, tranilast, and SB202190 reversed intracellular Ca^2+^ overload and H9c2 cardiomyocyte apoptosis induced by aconitine. These results suggested that aconitine promoted TRPV2 expression and PM metastasis through p38 MAPK signaling, thus inducing intracellular Ca^2+^ overload and cardiomyocyte apoptosis. Furthermore, TRPV2 is a potential molecular target for the treatment of aconitine poisoning.

## 1. Introduction

*Aconitum* species, containing aconitine, are widely used in the clinical treatment of rheumatism, arthritis, bruise, fracture, pain, and other diseases in China and other Asian countries because of their medicinal properties. However, due to their potential proarrhythmic effect, *Aconitum* and its related preparations are now restrictively used in the treatment of rheumatoid arthritis and some cardiovascular diseases [1]. As the main toxic ingredient and effective agent of *Aconitum*, aconitine is a natural diterpene alkaloid [2], which was reported to be an inducer of lethal ventricular arrhythmias through rapidly inhibiting or activating different ion channels on cardiac myocytes or conductive cells [3]. Although aconitine showed important biological activities in analgesia, diuresis, antitumor, antiasthmatic, anti-inflammatory, and other aspects [4, 5], its improper use can still lead to a high risk of serious toxic reactions, such as palpitation, vomiting, nausea, arrhythmia, shock, dizziness, hypotension, and coma [6]. Growing evidence showed that cardiotoxicity and neurotoxicity are the main toxic effects of aconitine [7]. According to previous studies, the mechanism of cardiotoxic effects may involve ion channel changes [8, 9], energy metabolism [10], oxidative damage [10], inflammation and apoptosis [11], and so on [12]. However, the cytotoxic signaling pathway of aconitine-induced cardiomyocyte injury remains to be further studied.

Transient receptor potential cation channel subfamily V member 2 (TRPV2) is a stretch-sensitive Ca^2+^ permeability channel. In myocardial tissue, TRPV2 was expressed in intercalated discs of the sarcomere and participated in the maintenance of appropriate electromechanical coupling and structure of the cardiomyocyte and myocardium [13]. It is also expressed in the cell pools of cardiomyocytes, mainly endoplasmic reticulum, and transferred to the sarcolemma under pathological conditions or stimulations, where it mediates a persistent Ca^2+^ influx and induces intracellular calcium overload [14]. Studies have shown that the p38 MAPK signaling pathway plays an important role in TRPV2 expression and transport to the plasma membrane (PM) because its activation can promote TRPV2 accumulation and transport to the PM [15, 16]. Meanwhile, it was reported that the arrhythmia induced by aconitine is related to the intracellular Ca^2+^ signal [17], and aconitine induces Ca^2+^ overload by activating the p38 MAPK signal, leading to arrhythmia and cardiomyocyte apoptosis [9]. p38 MAPK signaling plays an important role in cardiomyocyte differentiation, proliferation, apoptosis, inflammation, metabolism, and survival [18]. Studies have shown that p38 MAPK is related to cell cycle arrest of cardiomyocytes [19–21], which indicated that inhibition of p38 MAPK may be an effective strategy to enhance the proliferation of cardiomyocytes. The chronic activation of p38 MAPK was considered to be pathological and proapoptotic, and the inhibition of p38 MAPK activity was considered to be a potential therapy to alleviate acute injury of ischemic heart failure [22]. However, it is not clear whether aconitine-mediated cardiomyocyte Ca^2+^ overload and apoptosis are related to TRPV2 expression, PM metastasis, and p38 MAPK signal activation.

According to the above, here we hypothesized that aconitine could induce TRPV2-mediated Ca^2+^ influx through the p38 MAPK signal and thus promote cardiomyocyte apoptosis. The present study was designed to investigate this possibility *in vivo* which used the rat cardiomyocyte H9c2 cell line.

## 2. Materials and Methods

### 2.1. Cell Culture and Treatment

The rat cardiomyocyte H9c2 cells (#CRL-1446, ATCC) were cultured in the DMEM (Gibco, USA) with 10% FBS (Gibco, USA) and 0.1% penicillin-streptomycin solution (Sigma, USA) at 37°C in a 5% CO_2_ humidified incubator. Aconitine (content ≥ 98%) was purchased from the National Institute for the Control of Pharmaceutical and Biological Products (China). H9c2 cells were treated with different dosages of aconitine (0, 0.25, 0.5, and 1.0 *μ*M) for 24 h.

TRPV2 siRNA and negative siRNA were obtained from Shanghai GenePharma Co., Ltd., and transfected into H9c2 cells with a final concentration of 10 nM for 6 h by Lipofectamine^®^ 2000 (Invitrogen, USA) according to the manufacturer's protocols. Tranilast (Sigma, USA) was used to inhibit the activation of TRPV2 at a dosage of 75 *μ*M. SB202190 (Sigma, USA) was used to inhibit the activation of p38 at a dosage of 10 *μ*M.

### 2.2. Flow Cytometry

Flow cytometry assay was used to measure the cell apoptosis rate according to the previous report [23]. The apoptotic cells were double-labeled with annexin V-FITC and PI using an annexin V-FITC/PI apoptosis detection kit (Beyotime Biotechnology, China). H9c2 cells in each group were harvested and resuspended. The H9c2 cells were washed in cold sterile PBS, pelleted, counted (to determine the cell number), and resuspended in 1X annexin binding buffer at a concentration of 1 × 10^5^/100 *µ*L. Subsequently, the cells were incubated for 30 minutes at room temperature in the dark with FITC annexin V and propidium iodide (PI, 100 *µ*g/mL) and then further diluted with 400 *µ*L 1X annexin binding buffer. Then, the fluorescence intensity of the cells was quantified by using a flow cytometer (Accuri C6, BD Biosciences, San Jose, CA) using fluorescence emission at 530 nm (FL1) and >575 nm (FL3). Single color stains for FITC annexin and PI and unstained cells were included in all experiments as positive and negative controls.

### 2.3. Measurements of Intracellular Ca^2+^ Variation

Intracellular Ca^2+^ concentration variations were detected using the fluorimetric assay with Fura-2AM (a ratiometric probe for intracellular Ca^2+^) as essentially described [24]. The changes of intracellular Ca^2+^ were evaluated by fluorescence (510 nm) emission ratio at excitations at 340 and 380 nm, which can directly reflect the intracellular calcium content. In brief, the H9c2 cells were suspended in the buffer without Ca^2+^, and the basic fluorescence level was recorded; then, Ca^2+^ was applied at 2 mM leading to calcium influx through opened membrane calcium channels (control calcium level) after 20 s. In order to detect the influence of aconitine and p38 MPAK/TRPV2 inhibitors on the intracellular calcium content, they were added into the resuspended cells just before the beginning of the measurement, then each group of H9c2 cells was resuspended in buffer solution containing 2 mM Ca^2+^, and their fluorescence levels were recorded. To calculate the effect of inhibitors to aconitine, the normalized Ca^2+^ influx in the absence of aconitine and the channel activity at 2 mM Ca^2+^ are used as reference points.

### 2.4. Quantitative Reverse Transcription Polymerase Chain Reaction (qRT-PCR)

The performance of the qRT-PCR assay followed the methods of Peng et al. with some modification [25]. Total RNA was extracted from H9c2 cells using TRIzol reagent (Invitrogen, USA) and then reverse transcribed using a PrimeScript RT reagent kit (Takara Biotechnology Co., Ltd.), following the manufacturer's instructions (with the temperature protocol of 37°C for 15 min and 85°C for 5 sec). qRT-PCR was carried out using SYBR Real-Time PCR Master Mix (Takara Biotechnology Co., Ltd.) on an ABI 7500 Real-Time PCR System (Applied Biosystems, USA). The thermocycling conditions were as follows: initial denaturation at 95°C for 10 sec, followed by 40 cycles of 95°C for 10 sec and 60°C for 30 sec. The mRNA level was normalized to GAPDH, and the relative levels were calculated by the 2^−ΔΔCq^ method [26]. The primer sequences used were as follows: rat TRPV2, forward: 5′- GCTGGCTGAACCTGCTTTAC-3′, reverse: 5′-CTACAGCAAAGCCGAAAAGG-3′; GAPDH, forward: 5′-GACATGCCGCCTGGAGAAAC-3′, reverse: 5′- AGCCCAGGATGCCCTTTAGT-3'.

### 2.5. Western Blotting

Western blotting was used to examine the expression levels of proteins in this study; the method followed the methods of Peng et al. with some modifications [25]. Each group of H9c2 cells was harvested and lysed in RIPA buffer with protease inhibitors (Invitrogen, USA), and the protein concentrations were determined by the Pierce BCA assay (Invitrogen, USA), according to the manufacturer's protocols. Then, the proteins in lysates (40 ng of each sample) were separated by an SDS-PAGE and subsequently transferred onto PVDF membranes. The membranes were blocked with 5% nonfat milk for 1 h at room temperature and incubated with primary antibodies at 4°C overnight. Expression levels of the proteins of interest were analyzed using primary antibodies against the inhibitor of Bcl-2 (1 : 1000, CST, USA), Bax (1 : 1000, CST, USA), cleaved caspase-3 (1 : 1000, CST, USA), p38 (1 : 1000, CST, USA), p-p38 (1 : 1000, CST, USA), and TRPV2 (1 : 1000, Abcam, UK). Membranes were rinsed three times with 1X Tris-buffered saline with 0.5% Tween 20 (TBST) and then incubated with the anti-rabbit IgG (1 : 2000, Abcam, UK) horseradish peroxidase-conjugated secondary antibody for 1 h at room temperature. Membranes were rinsed three times with TBST and visualized using an ECL kit (Bio-Rad Laboratories Inc.). The protein bands were quantified using ImageJ software (version 1.52a, National Institutes of Health), and *β*-actin (1 : 1000, CST, USA) was used as a loading control. Each experiment was performed in triplicate.

### 2.6. Statistical Analysis

All the data are presented as the mean ± SEM. Differences between two or multiple groups were evaluated using a one-way ANOVA or two-way ANOVA followed by Bonferroni post hoc test. Statistical analyses were performed by GraphPad Prism 7.0 software (GraphPad Software Inc.). *P* < 0.05 was considered to indicate a statistically significant difference.

## 3. Results

### 3.1. Aconitine Promotes H9c2 Cardiomyocyte Apoptosis and Increases Ca^2+^ Influx

To detect the influence of aconitine on H9c2 cardiomyocyte, H9c2 cells were treated by aconitine at different dosages of 0, 0.25, 0.5, and 1.0 *μ*M for 24 h, and then the cell apoptosis and intracellular Ca^2+^ were measured. As the results show, aconitine induced obvious H9c2 cell apoptosis at a lower dose of 0.25 *μ*M, and the effect of aconitine on H9c2 cardiomyocyte apoptosis was dose dependent (Figures 1(a) and 1(b)). The levels of apoptosis-related proteins were carried out by western blotting (Figure 1(c)); the results showed that the expression of antiapoptotic protein Bcl-2 in H9c2 cells was reduced by aconitine at a dose-dependent manner, while the expressions of proapoptotic proteins Bax and cleaved caspase-3 were upregulated by aconitine at a dose-dependent manner (Figure 1(d)). In addition, aconitine obviously induced a Ca^2+^ influx which led to a significant intracellular Ca^2+^ overload of H9c2 cardiomyocytes in a dose-dependent manner (Figure 1(e)). These results indicated that aconitine could promote apoptosis by inducing intracellular Ca^2+^ overload.

### 3.2. Aconitine Activates the p38 MAPK Signal and Promotes TRPV2 PM Translocation

In order to further study the mechanism of aconitine on H9c2 cardiomyocyte apoptosis, the expressions of p38 MAPK and TRPV2 were determined. As shown in Figure 2(a), with the increase of the dosage of aconitine, there was a significant upregulation of the expression of p-p38, which was the activated form of p38 MAPK. For TRPV2, the results showed that both expression of TRPV2 mRNA and total TRPV2 protein level in H9c2 cardiomyocytes were all stimulated by aconitine in a dose-dependent manner (Figures 2(b) and 2(c)). Furthermore, aconitine not only induced the accumulation of TRPV2 in H9c2 cardiomyocytes but also promoted TRPV2 transfer to the PM which was established by increasing the cellular membrane expression of TRPV2 and the ratio between membrane TRPV2 and total TRPV2 (Figure 2(c)). These results implied that aconitine could activate the p38 MAPK signaling pathway and promote the expression and PM translocation of TRPV2.

### 3.3. Aconitine Promotes Ca^2+^ Influx by Upregulating TRPV2 Expression

To verify whether aconitine induced Ca^2+^ influx by promoting TRPV2 expression and PM transfer, siTRPV2 and specific TRPV2 inhibitor tranilast (TL) were used to inhibit TRPV2 expression and function. The results showed that TL had no obvious influence on the expression level of TRPV2, both mRNA and protein, which indicated TL could not inhibit the expression of TRPV2 but can inhibit the activation of TRPV2, while siTRPV2 significantly decreased the expression of TRPV2 mRNA and protein stimulated by aconitine (1.0 *μ*M) (Figures 3(a)–3(c)). Importantly, from the results of the Fura-2AM fluorimetric assay, there was a significant decrease of intracellular Ca^2+^ both in TL- and siTRPV2-treated groups compared with aconitine treated only (Figure 3(d), *P* < 0.001 compared with the 1.0 *μ*M aconitine treatment group), which indicated that TL has no obvious influence on TRPV2 expression but inhibits the activation of TRPV2, and TRPV2 inhibition by TL and siTRPV2 could reverse the Ca^2+^ influx induced by aconitine. These results suggested that the Ca^2+^ influx induced by aconitine was partly depended on the expression and activation of TRPV2.

### 3.4. Aconitine Promotes TRPV2 Transfer to the PM by Activating p38 MAPK Signaling

To detect whether aconitine promoted TRPV2 expression and PM translocation through p38 MAPK signaling, the p38 MAPK inhibitor SB202190 (SB) was used to inhibit the activation of p38 MAPK. As the results show, SB could effectively downregulate both mRNA and protein expression of TRPV2 stimulated by aconitine (1.0 *μ*M) (Figures 4(a)–4(c)). Meanwhile, SB obviously inhibited the activation of p38 MAPK induced by aconitine (Figures 4(b) and 4(c)). In addition, the PM translocation of TRPV2 induced by aconitine was obviously reduced by SB (Figures 4(b) and 4(c)), and upregulated intracellular Ca^2+^ stimulated by aconitine was reversed by SB as well (Figure 4(e)). These results indicated that aconitine could promote TRPV2 expression and PM transfer through activating p38 MAPK signaling.

### 3.5. p38 MAPK Inhibitor and TRPV2 Inhibitor Inhibit Aconitine-Induced Intracellular Ca^2+^ Overload and Cardiomyocyte Apoptosis

To further verify whether aconitine promoted TRPV2 expression and PM translocation through the p38 MAPK signal, thus mediating intracellular Ca^2+^ overload and inducing H9c2 cardiomyocyte apoptosis, SB and TL were used to inhibit the activation of p38 MAPK and TRPV2, respectively. As shown in Figures 5(a) and 5(b), both SB and TL alleviated the cell apoptosis induced by aconitine (1.0 *μ*M). SB downregulated the expression of cleaved caspase-3, p-p38, and membrane TRPV2 induced by aconitine, while TL just reduced the expression of cleaved caspase-3 and membrane TRPV2 significantly but had no obvious influence on the expression of TRPV2 (Figures 5(c) and 5(d)). In addition, both SB and TL reversed the Ca^2+^ influx promoted by aconitine (Figure 5(e)). These results suggested that p38 MAPK activation-induced TRPV2 expression and PM transfer played an important role in aconitine-induced H9c2 cardiomyocyte Ca^2+^ overload and apoptosis.

## 4. Discussion

*Aconitum*, as a world-famous medicinal plant, has been used for more than 2000 years. However, aconitine, as the main effective component of *Aconitum*, is a diterpenoid alkaloid with severe cardiovascular toxicity, which often induced tachyarrhythmia and hypotension and led to high mortality [27, 28]. Previous studies have shown that aconitine has obvious cytotoxicity on cardiomyocytes, which can induce cardiomyocyte injury through various ways, such as BNIP3-dependent mitophagy and TNF-*α*/NLRP3 signal transduction [11], Notch1-mediated histone demethylation of HCN4 [29], mitochondrial pathway [30], p38 MAPK signal, and Ca^2+^ overload [9]. In the present study, we demonstrated that aconitine could induce H9c2 cardiomyocyte apoptosis and Ca^2+^ influx in a dose-dependent manner (Figure 1), and the mechanism might be related to the activation of TRPV2 and p38 MAPK (Figure 2).

Growing evidence showed that the arrhythmia induced by aconitine is related to the activity of various ion channels, such as Na^+^ channel, Ca^2+^ channel, and K^+^ channel [31, 32]; among them, intracellular Ca^2+^ arrhythmia is most often reported to be related to the cardiotoxicity of aconitine [8, 9, 17, 33]. TRPV2 is a member of the TRPV channel family in the cardiovascular system and peripheral system and acts as a stretch-sensitive calcium permeability channel, and its plasma membrane translocation and activation lead to the sustained increase of intracellular Ca^2+^ [13]. TRPV2 is highly selective for Ca^2+^ and can be activated by lipids [34]. Under pathological conditions, the activation of TRPV2 mediates abnormal Ca^2+^ influx, thus accelerating disease progression [35], which is considered as a therapeutic target for cardiovascular diseases [13, 36]. Previous report has shown that inhibition of TRPV2 expression and intracellular Ca^2+^ overload plays an important role in maintaining cardiomyocyte activity and cardiac function [37]. The results of this study showed that both TRPV2 inhibitor tranilast and TRPV2 knockdown by siTRPV2 could reverse the Ca^2+^ influx stimulated by aconitine (Figure 3). Previous studies have revealed that the activation of the p38 MAPK signal could promote the expression and PM translocation of TRPV2 [15, 16], and the p38 MAPK signal could be activated by aconitine [9]. The present results showed that p38 MAPK inhibitor SB202190 reduced the expression and PM transfer of TRPV2 induced by aconitine, as well as Ca^2+^ influx (Figure 4), which indicated that aconitine could induce TRPV2-mediated Ca^2+^ influx by activating the p38 MAPK signal. Furthermore, tranilast and SB202190 reduced the H9c2 cardiomyocyte apoptosis stimulated by aconitine (Figure 5). These results suggested that aconitine-induced H9c2 cell apoptosis was partly depended on TRPV2-mediated intracellular Ca^2+^ overload promoted by p38 MAPK activation.

In summary, the effect of aconitine on cardiomyocytes was detected by *in vivo* assays in the present study, and results showed that aconitine promoted intracellular Ca^2+^ overload and cell apoptosis of H9c2 cardiomyocytes in a dose-dependent manner. Furthermore, aconitine promoted TRPV2 expression and PM metastasis through p38 MAPK signaling, thus inducing apoptosis mediated by intracellular calcium overload. These results indicated that TRPV2 may be a potential molecular target to treat aconitine poisoning and protect cardiac function.

## Figures and Tables

**Figure 1:** Influence of aconitine on apoptosis and Ca^2+^ influx of cardiomyocytes. (a, b) The rate of cell apoptosis was measured by flow cytometry. (c, d) The expressions of apoptosis-related proteins, Bcl-2, Bax, and cleaved caspase-3, were detected by western blotting. (e) The level of Ca^2+^ influx in each group was shown by the normalized ratio of 340/380. NC: negative control.  ^*∗*^^*∗*^*P* < 0.01,  ^*∗*^^*∗*^ ^*∗*^*P* < 0.001, and  ^*∗*^^*∗*^ ^*∗*^^*∗*^*P* < 0.0001 vs. the NC group.

**Figure 2:** The effect of aconitine on p38 MAPK signaling and TRPV2 expression. (a) The expressions of p38 and p-p38 in each group. (b) The level of TRPV2 mRNA was measured by qRT-PCR. (c) The expressions of total TRPV2 and membrane TRPV2. NC: negative control; t-TRPV2: total TRPV2; m-TRPV2: membrane TRPV2.  ^*∗*^*P* < 0.05,  ^*∗*^^*∗*^ ^*∗*^*P* < 0.001, and  ^*∗*^^*∗*^ ^*∗*^^*∗*^*P* < 0.0001 vs. the NC group.

**Figure 3:** Aconitine induces intracellular Ca^2+^ overload by activating TRPV2. (a) The expression level of TRPV2 mRNA. (b, c) The protein expressions of TRPV2 and m/t-TRPV2. (d) The intracellular Ca^2+^ level in each group. NC: negative control; MC: model control; TL: tranilast; siTRPV2: siRNA of TRPV2; t-TRPV2: total TRPV2; m-TRPV2: membrane TRPV2.  ^*∗*^*P* < 0.05,  ^*∗*^^*∗*^ ^*∗*^*P* < 0.001, and  ^*∗*^^*∗*^ ^*∗*^^*∗*^*P* < 0.0001 vs. the NC group; ^###^*P* < 0.001 and ^####^*P* < 0.0001 vs. the MC group.

**Figure 4:** Aconitine promotes TRPV2 expression and PM translocation by activating p38 MAPK signaling. (a) The expression level of TRPV2 mRNA. (b, c) The protein expressions of p38, p-p38, and TRPV2. (d) The intracellular Ca^2+^ level in each group. NC: negative control; MC: model control; SB: SB202190; t-TRPV2: total TRPV2; m-TRPV2: membrane TRPV2.  ^*∗*^*P* < 0.05 and  ^*∗*^^*∗*^ ^*∗*^^*∗*^*P* < 0.0001 vs. the NC group; ^##^*P* < 0.01, ^###^*P* < 0.001, and ^####^*P* < 0.0001 vs. the MC group.

**Figure 5:** p38 MAPK inhibitor and TRPV2 inhibitor inhibit aconitine-induced intracellular Ca^2+^ overload and apoptosis. (a, b) The cell apoptosis rate of cardiomyocytes. (c, d) The protein expressions of cleaved caspase-3, p-p38, and m-TRPV2. (e) The intracellular Ca^2+^ content level in each group. NC: negative control; MC: model control; SB: SB202190; TL: tranilast; t-TRPV2: total TRPV2; m-TRPV2: membrane TRPV2.  ^*∗*^*P* < 0.05,  ^*∗*^^*∗*^*P* < 0.01,  ^*∗*^^*∗*^ ^*∗*^*P* < 0.001, and  ^*∗*^^*∗*^ ^*∗*^^*∗*^*P* < 0.0001 vs. the NC group; ^##^*P* < 0.01, ^###^*P* < 0.001, and ^####^*P* < 0.0001 vs. the MC group.

## Data Availability

The datasets used and/or analyzed during the current study are available from the corresponding author upon reasonable request.

## References

[1] Ma L.-Q., Yu Y., Chen H. (2018). Sweroside alleviated aconitine-induced cardiac toxicity in H9c2 cardiomyoblast cell line. *Frontiers in Pharmacology*.

[2] Chan T. Y. K. (2012). Aconitum alkaloid content and the high toxicity of aconite tincture. *Forensic Science International*.

[3] Zhang F., Cai L., Zhang J., Qi X., Lu C. (2018). Aconitine-induced cardiac arrhythmia in human induced pluripotent stem cell-derived cardiomyocytes. *Experimental and Therapeutic Medicine*.

[4] Borcsa B., Widowitz U., Csupor D., Forgo P., Bauer R., Hohmann J. (2011). Semisynthesis and pharmacological investigation of lipo-alkaloids prepared from aconitine. *Fitoterapia*.

[5] Tang L., Gong Y., Lv C., Ye L., Liu L., Liu Z. (2012). Pharmacokinetics of aconitine as the targeted marker of Fuzi (Aconitum carmichaeli) following single and multiple oral administrations of Fuzi extracts in rat by UPLC/MS/MS. *Journal of Ethnopharmacology*.

[6] Lin C.-C., Chan T. Y. K., Deng J.-F. (2004). Clinical features and management of herb-induced aconitine poisoning. *Annals of Emergency Medicine*.

[7] Bisset N. G. (1981). Arrow poisons in China. part ii. aconitum -botany, chemistry, and pharmacology. *Journal of Ethnopharmacology*.

[8] Fu M., Wu M., Wang J.-F., Qiao Y.-J., Wang Z. (2007). Disruption of the intracellular Ca^2+^ homeostasis in the cardiac excitation-contraction coupling is a crucial mechanism of arrhythmic toxicity in aconitine-induced cardiomyocytes. *Biochemical and Biophysical Research Communications*.

[9] Sun G.-b., Sun H., Meng X.-b. (2014). Aconitine-induced Ca^2+^ overload causes arrhythmia and triggers apoptosis through p38 MAPK signaling pathway in rats. *Toxicology and Applied Pharmacology*.

[10] Zhao Y., Bu Q., Zhou Y. (2010). Mechanism study of Aconitum-induced neurotoxicity in PC12 cells: involvement of dopamine release and oxidative damage. *Neurotoxicology*.

[11] Peng F., Zhang N., Wang C. (2020). Aconitine induces cardiomyocyte damage by mitigating BNIP3-dependent mitophagy and the TNF*α*-NLRP3 signalling axis. *Cell Proliferation*.

[12] Sangiorgi G., Mauriello A., Bonanno E. (2006). Pregnancy-associated plasma protein-A is markedly expressed by monocyte-macrophage cells in vulnerable and ruptured carotid atherosclerotic plaques. *Journal of the American College of Cardiology*.

[13] Iwata Y., Matsumura T. (2019). Blockade of TRPV2 is a novel therapy for cardiomyopathy in muscular dystrophy. *International Journal of Molecular Sciences*.

[14] Entin-Meer M., Keren G. (2020). Potential roles in cardiac physiology and pathology of the cation channel TRPV2 expressed in cardiac cells and cardiac macrophages: a mini-review. *American Journal of Physiology-Heart and Circulatory Physiology*.

[15] Liu J., Zhao Z., Wen J. (2019). TNF‐*α* differently regulates TRPV2 and TRPV4 channels in human dental pulp cells. *International Endodontic Journal*.

[16] Ma W., Li C., Yin S. (2015). Novel role of TRPV2 in promoting the cytotoxicity of H2O2-mediated oxidative stress in human hepatoma cells. *Free Radical Biology and Medicine*.

[17] Zhou Y.-h., Piao X.-m., Liu X. (2013). Arrhythmogenesis toxicity of aconitine is related to intracellular Ca^2+^ signals. *International Journal of Medical Sciences*.

[18] Ruiz M., Coderre L., Allen B. G., Des Rosiers C. (2018). Protecting the heart through MK2 modulation, toward a role in diabetic cardiomyopathy and lipid metabolism. *Biochimica et Biophysica Acta (BBA)-Molecular Basis of Disease*.

[19] Engel F. B., Hsieh P. C. H., Lee R. T., Keating M. T. (2006). FGF1/p38 MAP kinase inhibitor therapy induces cardiomyocyte mitosis, reduces scarring, and rescues function after myocardial infarction. *Proceedings of the National Academy of Sciences*.

[20] Engel F. B., Schebesta M., Duong M. T. (2005). p38 MAP kinase inhibition enables proliferation of adult mammalian cardiomyocytes. *Genes & Development*.

[21] Engel F. B., Schebesta M., Keating M. T. (2006). Anillin localization defect in cardiomyocyte binucleation. *Journal of Molecular and Cellular Cardiology*.

[22] Marber M. S., Rose B., Wang Y. (2011). The p38 mitogen-activated protein kinase pathway-A potential target for intervention in infarction, hypertrophy, and heart failure. *Journal of Molecular and Cellular Cardiology*.

[23] Ji H., Xiao F., Li S., Wei R., Yu F., Xu J. (2020). GRP78 effectively protect hypoxia/reperfusion-induced myocardial apoptosis via promotion of the Nrf2/HO-1 signaling pathway. *Journal of Cellular Physiology*.

[24] Habes C., Weber G., Goupille C. (2019). Sulfated glycoaminoglycans and proteoglycan syndecan-4 are involved in membrane fixation of LL-37 and its pro-migratory effect in breast cancer cells. *Biomolecules*.

[25] Peng J., Jiang J., Wang H., Feng X., Dong X. (2020). miR-199a-3p Suppresses cervical epithelial cell inflammation by inhibiting the HMGB1/TLR4/NF-*κ*B pathway in preterm birth. *Molecular Medicine Report*.

[26] Livak K. J., Schmittgen T. D. (2001). Analysis of relative gene expression data using real-time quantitative PCR and the 2^−ΔΔCT^ method. *Methods*.

[27] Tai Y.-T., Lau C.-P., Young K., But P. P.-H. (1992). Cardiotoxicity after accidental herb-induced aconite poisoning. *The Lancet*.

[28] Chan T. Y. K. (2009). Aconite poisoning. *Clinical Toxicology*.

[29] Zhou W., Qiu L.-z., Liu H., Deng H.-F., Yue L.-X., Gao Y. (2020). Notch1-mediated histone demethylation of HCN4 contributes to aconitine-induced ventricular myocardial dysrhythmia. *Toxicology Letters*.

[30] Gao X., Zhang X., Hu J. (2018). Aconitine induces apoptosis in H9c2 cardiac cells via mitochondria-mediated pathway. *Molecular Medicine Reports*.

[31] Wu J., Wang X., Chung Y. Y. (2017). L-type calcium channel inhibition contributes to the proarrhythmic effects of aconitine in human cardiomyocytes. *PloS One*.

[32] Zhao Z., Yin Y., Wu H. (2013). Arctigenin, a potential anti-arrhythmic agent, inhibits aconitine-induced arrhythmia by regulating multi-ion channels. *Cellular Physiology and Biochemistry*.

[33] Zhang S.-W., Liu Y., Huang G.-Z., Liu L. (2007). Aconitine alters connexin43 phosphorylation status and [Ca^2+^] oscillation patterns in cultured ventricular myocytes of neonatal rats. *Toxicology in Vitro*.

[34] Guéguinou M., Felix R., Marionneau-Lambot S. (2021). Synthetic alkyl-ether-lipid promotes TRPV2 channel trafficking trough PI3K/Akt-girdin axis in cancer cells and increases mammary tumour volume. *Cell Calcium*.

[35] Rozenbaum Z., Cohen L., Bigelman E., Shacham Y., Keren G., Entin-Meer M. (2018). Downregulated expression of TRPV2 in peripheral blood cells following acute myocardial infarction is inversely correlated with serum levels of CRP and troponin I. *Cardiology*.

[36] Aguettaz E., Bois P., Cognard C., Sebille S. (2017). Stretch-activated TRPV2 channels: role in mediating cardiopathies. *Progress in Biophysics and Molecular Biology*.

[37] Li Y., Li Q., Zhang O. (2019). miR‐202‐5p protects rat against myocardial ischemia reperfusion injury by downregulating the expression of Trpv2 to attenuate the Ca^2+^ overload in cardiomyocytes. *Journal of Cellular Biochemistry*.

